# Performance assessment of solar tower collector based integrated system for the cogeneration of power and cooling

**DOI:** 10.1016/j.heliyon.2024.e39993

**Published:** 2024-10-30

**Authors:** Mohd Asjad Siddiqui, Ibrahim Alsaduni

**Affiliations:** a Department of Mechanical Engineering, Faculty of Engineering and Technology, Jamia Millia Islamia, New Delhi, 110025, India; b Department of Electrical Engineering, College of Engineering, Majmaah University, Al-Majmaah, 11952, Saudi Arabia

**Keywords:** S-CO_2_ power cycle, Absorption refrigeration cycle, Exergy, ORC, Solar power tower

## Abstract

Integrating solar energy systems is an essential measure in advancing worldwide sustainability objectives and offers a sustainable, environmentally friendly approach to reducing greenhouse gas emissions and pollutants. To this direction, the proposed system integrating solar tower collector, supercritical CO_2_, organic Rankine cycle, and single effect absorption refrigeration cycles shows potential as an efficient and sustainable solution for meeting energy and cooling demands. A detailed thermodynamic evaluation has been performed to gain valuable understanding of the energy and exergy performance, enabling the assessment of thermal and exergy efficiencies, exergy destructions, and heat losses. Results show that this study found the thermal efficiency of the proposed system to be 47.35 % for R245fa, 48.59 % for R123, and 52.32 % for toluene. In addition, the exergy efficiency was obtained at 40.99 % for R245fa, 42.41 % for R123, and 46.67 % when toluene is used as a working fluid. With all investigated working fluids of organic Rankine cycle, toluene achieved the highest thermal and exergy efficiency of the proposed power-cooling cogeneration system, while R245fa achieved the lowest energetic and exergetic performance. Among the various ORC working fluids investigated under operating conditions, toluene demonstrated the highest turbine power output (3202 kW), whereas R245fa exhibited the lowest turbine power output (2804 kW). The refrigeration output for all ORC working fluids studied was found to be 988.8 kW. Additionally, the primary contributor of exergy destruction rate in the proposed system was determined to be the solar tower receiver, contributing 73.24 %, 67.80 %, and 66.19 % to the total for the toluene, R123, and R245fa working fluids, respectively.

## 1 Introduction

Population and industry growth is going to create a challenge to meet rising energy demand, which needs higher energy generation. Combustion of conventional resources of energy, like oil, coal, and natural gas, dominates conventional power electricity production. Because of the scarcity of available energy and related greenhouse gas (GHG) emissions, it is critical to seek alternative energy sources that have a minimal impact on the ecosystem. The global distribution of GHG emissions by gas, depicted in Fig. 1 (a), indicates that carbon dioxide, the most abundant gas, accounts for a substantial majority of total emissions at 74.4 %. Furthermore, the figure illustrates that other greenhouse gases like methane (17.3 %), nitrous oxide (2.39 %), and F-gases (2.1 %) make a smaller but still significant contribution to global GHG emissions. It is noteworthy that the largest proportion of emissions by sector, approximately 73.2 %, is attributed to energy use, as indicated in Fig. 1 (b). Agriculture and land use also play a substantial role, accounting for nearly 18.4 % of emissions, while industry and waste contribute 5.2 % and 3.2 % respectively to the total emissions [1].

**Fig. 1:** The distribution of worldwide GHG emissions by (a) gas and (b) sector.

Energy from renewable sources, like wind, geothermal and solar energy are currently being investigated as potential replacements for conventional fossil fuels to tackle the previously mentioned problem. Solar energy has gained significant attention in the field of renewable energy due to its widespread availability and abundance, making it one of the most convenient and accessible sources of energy to utilize [2,3]. Additionally, it is the most efficient source of generating power and heat while also mitigating environmental impacts [4].

In recent decades, there has been considerable interest in optimizing the utilization of solar energy through the development of concentrating solar power technologies. Solar tower collector technology stands out among other concentrated solar power (CSP) technologies due to its ability to generate high temperatures, resulting in enhanced power cycle efficiency [5,6]. Kalogirou [7] studied the temperature range suitable for the operation of various solar thermal technologies, including parabolic trough collectors (60°C−500°C), solar dishes (100 °C–700 °C), and heliostat fields (150 °C–1500 °C).

According to Wang et al. [8], the performance of several cycles for central receiver system applications were designed and evaluated. The results indicated that the heliostat fields technique has the best performance, the most potential for scaling, and the most flexibility in terms of the temperature range compared to all high-temperature solar methods. Wu and Wang [9] initially developed the distributed energy system (DES) to provide electrical, thermal, and cooling energy in order to improve the stability of the energy supply. In addition, because It is placed near the consumer, it can efficiently reduce energy loss and boost efficiency by utilizing waste heat in a cascaded manner [10]. Moreover, distributed energy systems are designed to accommodate the distribution characteristics of energy from renewable sources, including solar and wind energy. Heat exchangers are a simple way to meet customers' heating needs in a distributed energy system. In contrast, the methods for producing power and providing cooling in these systems are inherently intricate and difficult to execute [11,12]. The integration of combined power and cooling (CPC) systems has become crucial for the effective implementation of DES applications due to the complex nature of these processes [13]. Consequently, CPC solutions have attracted significant interest and focus from both researchers and industry experts in recent years [14,15].

In the field of power generation, it is essential to investigate alternative approaches to the conventional steam Rankine cycle with the aim of improving efficiency and reducing the expenses associated with electricity production in power plants. One such promising solution is the supercritical carbon dioxide (s-CO_2_) power cycle, which presents several benefits aligned with sustainability goals [16]. It is recognized for its compact and simple design, making it easier to deploy and operate, while also delivering higher efficiency when compared to conventional Rankine cycles. The smaller equipment sizes enabled by this compact design lead to reductions in both capital and operational costs. Significantly, s-CO2 power cycles provide a lower compression work and higher thermal efficiency in comparison to conventional power cycles, as they utilize eco-friendly working fluids like supercritical carbon dioxide, which enhances heat transfer properties and energy conversion efficiency, thereby decreasing greenhouse gas emissions and promoting a more sustainable energy future [17,18]. Zhai et al. [19] conducted a comparative analysis on steam Rankine cycle, s-CO_2_ Brayton cycle, and air Brayton cycle. Their findings suggest that the s-CO_2_ Brayton cycle shows promise for efficiently harnessing solar energy across a wide range of temperatures from 250 to 1000 °C. The higher efficiency of the s-CO_2_ Brayton cycle compared to the other two cycles indicates its potential to convert a larger portion of thermal energy from concentrated solar power into useful work, ultimately enhancing overall system performance. Yilmaz et al. [20] designed a solar-based multigeneration system that integrates a s-CO_2_ Brayton cycle, transcritical Rankine cycle, multi-effect desalination unit, and PEM electrolyzer. Their findings indicate that the energetic and exergetic efficiency of the s-CO_2_ Brayton cycle is calculated at 16.61 % and 59.35 %, respectively.

The CPC system is being employed as a bottoming cycle to fully utilize traditional power cycle waste heat and an extremely effective way to use low-temperature heat sources such as solar and geothermal energy, and waste heat from industrial processes. Geothermal energy was used as a heat source in a cogeneration system designed by Parikhani et al. [21] based on the absorption power cycle for generating power and cooling simultaneously. It was discovered that, at a geothermal inlet temperature of 145 °C, the cycle achieves thermal and exergy efficiencies of 16.4 % and 28.95 %, respectively. An innovative configuration of the power-cooling system were proposed by Barkhordarian et al. [22] to use NH_3_-H_2_O as the working fluid and two evaporators for cooling at two different temperatures. According to the results of the simulation studies, the cycle obtained thermal and exergy efficiencies of 19 % and 38.97 % respectively, within the specified conditions. A solar-driven cogeneration system designed by Siddiqui et al. [23] developed an innovative power-cooling system that utilizes engine waste heat by combining the ORC with the ERC. The essential parameters and their impact on the performance of the system were investigated using various working fluids. Ventas et al. [24] introduced a dual double-effect absorption system that utilizes either solar or residual energy to generate both power and cooling simultaneously, with an ammonia/lithium nitrate mixture operating as the working fluid. At 132 °C generating temperature, the proposed system exhibits a thermal efficiency of 6.5 % and a coefficient of performance (COP) of 0.52.

Muye et al. [25] studied a cogeneration system driven by solar energy for power and cooling in a building, which incorporated an absorption refrigeration cycle and a biomass auxiliary system. In their study, the authors found that the scroll expander exhibited an efficiency range of 59 %–63 % per annum, whereas the system demonstrated a yearly efficiency range of 6 %–8 %. According to their conclusion, based on the system location and temperature of the evaporator, the annual solar contribution varies between 23 and 30 %. Perdichizzi et al. [26] analyzed a cogeneration system driven by solar energy to supply power and cooling. This system was developed to run in a specified mode in order to meet the hourly demands for both power and cooling. In their assessment, implementing the proposed method can significantly reduce fossil fuel usage during peak hours in summer and winter. Shaaban [27] proposed a modified integrated solar combined cycle to improve the overall performance of the investigated combined cycle with dual bottoming cycles.

Although there have been numerous studies on the performance analysis of combined power and cooling systems using traditional working fluids and various energy sources, very few researchers have focused on the impact of the specific type of energy source and system employed. The utilization of parabolic collectors for harnessing solar energy is widespread, but the superior performance of heliostat based systems makes it a compelling choice for capturing solar energy, which is the focus of the current research. Additionally, the heat transfer fluid used in this study was molten salt (60 % NaNO_3_ and 40 % KNO_3_), which is capable of reaching higher temperatures than oils and exhibits superior heat transfer properties compared to oils. Previous studies have not examined the performance of a solar-based cogeneration system that includes solar tower collectors as the primary movers, an s-CO_2_ and ORC cycles for power production, and single effect LiBr-H_2_O absorption chiller for cooling a specific building. In this study, a power-cooling system is thermodynamically investigated in terms of energy and exergy under steady-state conditions to meet the summer air conditioning demands. R123, R245fa, and toluene have been assessed as potential working fluids for the ORC and the best working fluid for the ORC is determined from the chosen fluids. When examining the performance of energy conversion systems, exergy analysis proves to be more informative. This is because it has the ability to identify the locations, magnitudes, and sources of thermodynamic inefficiencies within these systems. In this study, a comprehensive analysis of energy and exergy issues has been conducted. The evaluation of system output parameters, including cogeneration system efficiencies (thermal and exergy), power, and refrigeration outputs, for the components under different operating conditions has been examined. These include characteristics such as solar irradiation, heliostat field area, s-CO_2_ turbine inlet temperature, evaporator temperature, and condenser temperature of the ORC, among other factors.

Consequently, the goal of this study is to assess the thermodynamic modelling and exergetic analysis of a solar tower collector driven power-cooling cogeneration system. The sub-objectives follow:

• To develop a solar driven high-efficiency cogeneration system that meets the energy needs of buildings or applications requiring power and cooling in a sustainable and eco-friendly manner.
• Recovery of low-grade waste heat from the s-CO_2_ turbine exhaust is achieved using an ORC cycle and a LiBr-H_2_O based ARC cycle for generating power and cooling.
• A mathematical model is developed, and thermodynamic investigation is performed employing Engineering Equation Solver (EES) software to determine the optimal design variables and configuration to enhance the performance of the system from both energy and exergy perspectives under consideration [28].
• R123, R245fa, and toluene are assessed as potential working fluids for the ORC and the best working fluid for the ORC is determined from the chosen fluids.
• To perform a comprehensive parametric assessment by varying the significant parameters on achieving maximum thermal and exergetic performance of the proposed cogeneration system.
• To identify and reduce irreversibilities in system components in order to improve overall system performance by targeting weak spots that contribute to the highest exergy loss.

## 2 System description

The layout of the proposed cogeneration system for power and cooling in Fig. 2 demonstrates that the heat source is provided by the solar power tower, while the generation of electricity is carried out by the s-CO_2_ and ORC turbines. In contrast, a single-effect LiBr-H_2_O absorption chiller serve as the cooling system. In this system, we can observe that three cycles are employed, including the s-CO_2_ and ORC cycles as power generation units, and the ARC cycle for cooling. s-CO_2_ cycle waste heat is used to fulfil power and cooling demands, with a portion of it being used to generate electricity employing an ORC cycle, while another amount of it is used to cool by means of an absorption chiller. The integrated system comprises four subsystems: the solar tower collector, the s-CO_2_ cycle, the ORC cycle, and the ARC cycle.

**Fig. 2:** The proposed solar-powered cogeneration system for power and cooling.

### 2.1 Solar tower collector

The solar tower collector is widely recognized as a highly efficient technology for utilizing solar energy. Its distinctive design enables the concentration and capture of solar energy by employing a heliostat field and a central receiver. In this procedure, molten salt (60 % NaNO_3_ and 40 % KNO_3_) is employed as a heat transfer medium within the receiver tubes to transmit the solar energy. The selection of molten salt in this research is supported by its exceptional performance characteristics (as demonstrated in Table 1), specifically its elevated energy conversion rate. The HTF is moved to a receiver employing a HTF pump and collects heat from reflected radiation. It then effectively transmits the heat to the s-CO_2_ cycle fluid through a heat exchanger-1.

**Table 1:** Characteristics of HTF [29].

Parameter	Value
HTF	Molten salt
Density (kg m^−3^)	ρ=2090−0.636∗T(°C)
Thermal conductivity (W K^−1^ m^−1^)	$\lambda =0.443+1.9*10^{-4}*T\left({}^{\circ}C\right)$
Specific heat (kJ K^−1^ kg^−1^)	$c_{p}=1443+0.172*T\left({}^{\circ}C\right)$
Lower temperature limit (°C)	220
Upper temperature limit (°C)	600

### 2.2 Supercritical carbon-dioxide (s-CO_2_) cycle

In the s-CO_2_ cycle, the compressed working fluid CO_2_ (point 9) is heated by the high temperature CO_2_ from the s-CO_2_ turbine in the heat exchanger-2 (10–11). Furthermore, the CO_2_ is heated once more in heat exchanger-1 (11–4) by the high-temperature fluid from the solar tower collector. The high temperature CO_2_, upon leaving heat exchanger-1 (point 4), is directed into the turbine for expansion to generate useful work. Subsequently, the high temperature expanded fluid (point 5) is then directed into heat exchanger-2 to serve as a heat source for the ORC cycle. The high temperature fluid leaving heat exchanger-2 goes to the generator (point 7) after releasing heat through the recuperator (6–7), where it acts as a heat source for ARC cycle and then returns to the compressor (point 9) after releasing heat through the pre-cooler (8–9).

### 2.3 Organic Rankine cycle (ORC)

A heat exchanger (HE-2), an ORC turbine (T2), an ORC condenser (C1), and an ORC pump (P2) are all included in the Organic Rankine cycle, as depicted in Fig. 1. Organic fluid is heated in the heat exchanger (HE-2) of the ORC cycle (15–12) using high-temperature exhaust fluid from the s-CO_2_ turbine (5–6). Then, mechanical power is generated by the ORC-Turbine (12–13) using the heated organic fluid. The heated stream from the ORC turbine leaves and enters the condenser (point 13) and pumping back to the heat exchanger (HE-2) of the ORC.

### 2.4 Absorption refrigeration cycle (ARC)

In the ARC cycle, the CO_2_ fluid leaving the recuperator is transferred into the generator at point 7, working as a heat source for the ARC cycle and producing a cooling load in the evaporator. The heat generated by the generator is utilized to vaporize the water in the LiBr-H_2_O mixture and transfer it to the condenser (point 16). At this stage, condensation takes place in the condenser, leading to the production of a saturated liquid that exits from the condenser (point 17). Subsequently, upon throttling of the water, a low-temperature mixture of liquid and vapor is formed (point 18) and is directed towards the evaporator. The primary role of the evaporator is to meet the cooling requirements of the system. The vaporized water produced by the evaporator is carefully directed into the absorber (point 19). The vaporized water is absorbed by the Li-Br, resulting in a mixture of Li-Br and water. Subsequently, the mixture is directed to the solution heat exchanger at point 21 through pump 3. The solution heat exchanger efficiently increases the temperature of the mixture and directs it into the generator at point 22, thereby completing the cycle.

As stated in Table 1, the current study employed molten salt as a medium for heat transfer, which is comprised of a combination of 60 % NaNO_3_ and 40 % KNO_3_.

### 2.5 Selection of working fluids

Working fluid selection for ORC is crucial because the performance of the ORC system is entirely dependent on the working fluid. Because of this, it is necessary to choose the correct working fluid to increase thermal output and make the best possible use of waste heat, and for this reason, three different working fluids have been investigated for this study. Consequently, the selection of an organic fluid to be used in ORC should consider a few other characteristics in addition to the system-based thermal performance. These characteristics include flammability, toxicity, Global Warming Potential (GWP), and Ozone Depletion Potential (ODP). The critical temperature of a working fluid is the most significant characteristic to consider because it is responsible for determining the highest level of evaporation temperature achieved during the subcritical cycle. The working fluids with critical temperatures of 183.7 °C, 154.01 °C, and 318.6 °C have been selected for an investigation to design an ORC that can produce acceptable amounts of power. Fluids with a lower or higher critical temperature are not a suitable option because, in the case of a lower critical temperature, the turbine will not produce a large amount of power due to the limitation of a high heat rejection temperature in the condenser to utilize it in the absorption heat pump. Conversely, fluids with higher critical temperatures may be accompanied by potential design issues related to the thermal fluid. These factors mean that lower and higher critical temperature fluids are not excellent choices. Therefore, in light of the work accomplished by earlier researchers, we conduct an exhaustive analysis of a wide range of substances, taking into account their thermodynamic properties as well as other factors such as cost, stability, and so on, and we select R123, R245fa, and Toluene as the working fluids. The thermophysical characteristics of the selected fluids are mentioned in Table 2.

**Table 2:** Thermophysical characteristics of selected working fluids.

Refrigerant	R123	R245fa	Toluene
Chemical Formula	C_2_HCl_2_F_3_	C_3_F_5_H_3_	C_7_H_8_
Critical temperature (^o^C)	183.7	154.01	318.6
Critical pressure (kPa)	3668	3651	4126
Normal boiling point (^o^C)	27.78	15.18	110.6
Triple point Temperature (^o^C)	−107.2	−102.1	−94.97
Molecular Weight (kg/kmol)	152.9	134.04	92.14
Safety class	B1	B1	B3
ODP	0.02	0	0
GWP	77	1030	–

## 3 Modelling of solar tower collector

A power-cooling proposed cogeneration system powered by solar tower collectors, which includes the heliostat field and the molten salt central receiver. A variety of heat losses in the receiver can be calculated using the equations listed below, including the total amount of heat absorbed by the receiver.

The heat rate derived from solar irradiation is expressed as [30]:

(1) $${\dot{Q}}_{solar}=I*A_{field}$$

Where, *I* represents the solar irradiation $\left(W/m^{2}\right)$ and $A_{field}$ refers to the area of heliostat field ($m^{2})$.

The receiver's net energy balance can be expressed as follows [30].

(2) $${\dot{Q}}_{CR}={\dot{Q}}_{CR,abs}+{\dot{Q}}_{lost,CR}$$

The amount of heat absorbed by the molten salt as it flows through the receiver can be calculated as [31].

(3) $${\dot{Q}}_{CR,abs}={\dot{m}}_{ms}*C_{p}\left(T_{ms,out}-T_{ms,in}\right)$$

Where, ${\dot{m}}_{ms}$ & $C_{p}$ are the molten salt mass flow rate and specific heat, $T_{ms,in}$ & $T_{ms,out}$ are the molten salt inlet and outlet temperature.

The central receiver undergoes heat loss at a rate that is determined by the combined effects of emissive, convective, and reflective losses. The total loss calculated as follows [31]:

(4) $${\dot{Q}}_{lost,CR}=\underset{emissive\;losses}{\underbrace{{\dot{Q}}_{CR}*F_{r}*\chi }}+\underset{convective\;losses}{\underbrace{h_{c}*A_{ap}*\left(T_{r}-T_{o}\right)}}+\underset{reflective\;losses}{\underbrace{\varepsilon *\sigma *A_{ap}*F_{r}*\left({T_{r}}^{4}-{T_{o}}^{4}\right)}}$$

Where, $F_{r}$ represents the view factor, $h_{c}$ is the convective heat transfer coefficient, χ represents the reflectivity of the receiver surface, σ is the Stefan– Boltzmann constant, $A_{ap}$ is the aperture area and ε is the average emissivity. $T_{r}$ is used to denote the temperature of the receiver, while $T_{o}$ denotes the atmospheric temperature.

The temperature of receiver surface can be determined as [31]:

(5) $$\frac{{\dot{Q}}_{CR}}{F_{r}*A_{field}*C}=\frac{\left(T_{r}-T_{m}\right)}{\frac{d_{o}}{d_{i}*h_{ms}}+\frac{d_{o}}{2*k_{w}}\ln\;\left(\frac{d_{o}}{d_{i}}\right)}$$

Where, *C* represents the concentration ratio, $T_{m}$ denotes HTF mean temperature $d_{i}$ and $d_{o}$ are the tube diameters of inner and outer, $h_{ms}$ represents the coefficient of convection and $k_{w}$ denotes the tube thermal conductivity.

The energy efficiency of heliostat is determined as [30].

(6) $$\eta_{H}=\frac{{\dot{Q}}_{CR}}{{\dot{Q}}_{solar}}$$

The receiver's aperture area is determined as

(7) $$A_{ap}=\frac{A_{field}}{C}$$

The exergy rate derived from solar irradiation is expressed as [30].

(8) $${\dot{E}}_{x,solar}={\dot{Q}}_{solar}\left(1-\frac{T_{0}}{T_{sun}}\right)$$

Where, $T_{sun}$ denotes the apparent sun temperature

The exergy provided to the receiver is expressed as [30].

(9) $${\dot{E}}_{x,CR}={\dot{E}}_{x,CR,abs}+{\dot{E}}_{x,lost,CR}$$

(10) $${\dot{E}}_{x,CR,abs}={\dot{m}}_{ms}*C_{p}*\left[\left(T_{ms,out}-T_{ms,in}\right)-T_{0}\;\ln\left(\frac{T_{ms,out}}{T_{ms,in}}\right)\right]$$

(11) $${\dot{E}}_{x,lost,CR}={\dot{Q}}_{lost,CR}\left(1-\frac{T_{0}}{T_{r}}\right)$$

The exergetic efficiencies of heliostat field and receiver are expressed as [30]:

(12) $$\eta_{ex,H}=\frac{{\dot{E}}_{x,CR}}{{\dot{E}}_{x,solar}}$$

(13) $$\eta_{ex,CR}=\frac{{\dot{E}}_{x,CR,abs}}{{\dot{E}}_{x,CR}}$$

## 4 Thermodynamic modelling

The assumptions stated in this section form the basis for the energy and exergy analysis of the various components of the proposed solar tower collector power and cooling cogeneration system [30, 4, 15, 32).

• The proposed system is designed to operate in a steady state.
• The chemical exergy in the proposed cycle can be ignored since no chemical reactions take place. Additionally, the kinetic and potential energies are not considered.
• It is assumed that the turbines and pumps are adiabatic.
• ARC expansion and throttling valves are isenthalpic and pressure-reducing devices.
• The single-effect absorption system is capable of operating at its maximum cooling capability.
• No changes in the pressure owing to leaks or drops are considered during system operation
• For ARC and ORC, only the physical exergies of the LiBr-H_2_O fluid pair and the ORC fluid are taken into consideration.
• Saturated states are assumed at the condenser and evaporator outputs.

According to the assumptions used in the current work, the solar-driven cogeneration system for power and cooling in the city of Madinah, Kingdom of Saudi Arabia is situated at a latitude of 24.5°N and a longitude of 39.5°E, under precise sky circumstances, with an average relative humidity of 65 % and an ambient temperature of 15 °C. Table 3, Table 4 provide the input parameters used in the study of the proposed system.

**Table 3:** Constant operating conditions for the thermodynamic analysis of proposed cogeneration system in present study.

Constant parameters	Value
Atmospheric temperature (°C)	25 °C
Atmospheric pressure (kPa)	101.325
Aperture area ($A_{ap}$) $\left(m^{2}\right)$	12.5
Stefan–Boltzmann constant (σ) $\left(J/m^{2}sK^{4}\right)$	$5.6\times 10^{-8}$
Emissivity (ε)	0.8
Reflectivity (χ)	0.04
View factor ($F_{r}$)	0.8
Tube thickness (m)	0.00165
Inlet diameter of tube (m)	0.019
Sun temperature (K)	5778
Thermal efficiency of heliostat (%)	75
Inlet temperature of HTF (°C)	290
Isentropic efficiency of turbine (%)	95
Inlet pressure of turbine (kPa)	13000
Generator temperature (°C)	90
Solution heat exchanger effectiveness (%)	80
ARC condenser temperature (°C)	35
Temperature at the absorber (°C)	35

**Table 4:** Variable operating parameters for the thermodynamic modelling of proposed system in present study.

Variable parameters	Default value	Investigated range
Solar Irradiation ($W/m^{2}$)	1000	900–1100
Heliostat field area ($m^{2}$)	10000	9000–11000
s-CO_2_ turbine inlet temperature (°C)	500	450–750
ORC Condenser Temperature (°C)	35	30–42
Evaporator temperature (K)	278	270–286

The application of the first law of thermodynamics is utilized to perform an energy evaluation of the system's constituents. General equations for mass and energy balance can be formulated as follows [15,33].

(14) $$\Sigma {\dot{m}}_{in}-\Sigma {\dot{m}}_{out}=0$$

(15) $$\Sigma \dot{Q}-\Sigma \;\dot{W}=\Sigma {\left(\dot{m}h\right)}_{out}-\Sigma {\left(\dot{m}h\right)}_{in}$$

Where $\dot{Q}$ for heat transfer rate, $\dot{W}$ for fuel, $\dot{m}$ for rate of mass flow, h for specific enthalpy, and in and out subscript stands for inlet and outlet of control volume, respectively.

The exergy approach, based on the second law of thermodynamics, is a useful method for identifying irreversibility and analyzing thermodynamic inefficiencies in a system. Because each portion has thermodynamic irreversibility, the exergy modelling approach is used to assess the output for recovering low-temperature waste heat from the environment. Consider T_0_ and P_0_ to be the ambient temperature and pressure as the defined dead reference state.

According to the assumptions, variations in potential and kinetic energy are not taken into consideration. This results in ${\dot{E}}_{x}$ being treated as the entire exergy of both physical and chemical exergy, as seen in the following equation:

(16) $${\dot{E}}_{x}={\dot{E}}_{x}^{ph}+{\dot{E}}_{x}^{ch}$$

The chemical exergy can be disregarded in the suggested cycle due to the absence of chemical reactions. Consequently, at any given instant during a state, the exergy ${\dot{E}}_{i}$ equals the physical exergy ${\dot{E}}_{x}^{ph}$ that is obtainable [34].

(17) $${\dot{E}}_{i}={\dot{E}}_{x}^{ph}={\dot{m}}_{i}\left[\left({h_{i}-h}_{0}\right)-T_{0}\left({s_{i}-s}_{0}\right)\right]$$

The exergy balance equation for an open thermodynamic system is shown below [8]:

(18) $${\dot{E}}_{x}=\Sigma \left({\dot{E}}_{in}\right)-\Sigma \left({\dot{E}}_{out}\right)$$

(19) $${\dot{E}}_{x,heat}-\Sigma \dot{W}+\Sigma {\dot{m}}_{in}e_{x_{in}}-\Sigma {\dot{m}}_{out}e_{x_{out}}-{\dot{E}}_{x,D}=0$$

Where $\dot{W}$ denotes work input, $\dot{m}$ denotes mass flow rate, and ${\dot{E}}_{x,D}$ denotes the rate of exergy destruction, and in and out signify input and output conditions, respectively.

The exergy related to heat transfer $\dot{Q}$ from a constant temperature T source can be described as [33]

(20) $${\dot{E}}_{x,heat}=\sum {\left(\dot{Q}\left(1-\frac{T_{0}}{T}\right)\right)}_{in}+\sum {\left(\dot{Q}\left(1-\frac{T_{0}}{T}\right)\right)}_{out}$$

The energy and exergy balancing equations in each component are formulated by applying the above general equations to the proposed solar-based cogeneration system for power and cooling, and they are shown in Table 5.

**Table 5:** Energy and exergy balances equations for each component of a solar-driven power-cooling cogeneration system.

Component		Balance Equations
Heat Exchanger (HE1)	Energy balance	${\dot{m}}_{ms}\;\left(h_{1}-h_{2}\right)={\dot{m}}_{CO2}\;\left(h_{4}-h_{11}\right)$
	Exergy balance	${\dot{E}}_{x,D,HE1}={\dot{m}}_{ms}e_{x,1}+{\dot{m}}_{CO2}e_{x,11}-{\dot{m}}_{CO2}e_{x,4}-{\dot{m}}_{ms}e_{x,2}$
Molten salt pump (P1)	Energy balance	${\dot{W}}_{P1}={\;\dot{m}}_{ms}\;\left(h_{3}-h_{2}\right)$
	Exergy balance	${\dot{E}}_{x,D,P1}$*=*${\dot{m}}_{ms}\left(e_{x,2}-e_{x,3}\right)+{\dot{W}}_{P1}$
s-CO_2_ turbine (T1)	Energy balance	${\dot{W}}_{T1}={\dot{m}}_{CO2}\;\left(h_{4}-h_{5}\right)$
	Exergy balance	${\dot{E}}_{x,D,T1}={\dot{m}}_{CO2}e_{x,4}-{\dot{W}}_{T1}-{\dot{m}}_{CO2}e_{x,5}$
Heat Exchanger (HE2)	Energy balance	${\dot{Q}}_{HE2}={\dot{m}}_{12}\;\left(h_{12}-h_{15}\right)={\dot{m}}_{CO2}\;\left(h_{5}-h_{6}\right)$
	Exergy balance	${\dot{E}}_{x,D,HE2}={\dot{m}}_{CO2}\left(e_{x,5}-e_{x,6}\right)+{\dot{m}}_{12}\left(e_{x,15}-e_{x,12}\right)$
Recuperator	Energy balance	${\dot{m}}_{CO2}\left(h_{11}-h_{10}\right)={\dot{m}}_{CO2}\left(h_{6}-h_{7}\right)$
	Exergy balance	${\dot{E}}_{x,D,rec}={\dot{m}}_{CO2}\left(e_{x,10}-e_{x,11}\right)+{\dot{m}}_{CO2}\left(e_{x,6}-e_{x,7}\right)$
Pre-cooler	Energy balance	${\dot{Q}}_{pc}={\dot{m}}_{CO2}(h_{8}-h_{9}$)
	Exergy balance	${\dot{E}}_{x,D,pc}={\dot{m}}_{8}e_{x,8}-{\dot{m}}_{9}e_{x,9}$
Compressor	Energy balance	${\dot{W}}_{C}={\dot{m}}_{CO2}\left(h_{10}-h_{9}\right)$
	Exergy balance	${\dot{E}}_{x,D,C}={\dot{W}}_{C}+{\dot{m}}_{9}e_{x,9}-{\dot{m}}_{10}e_{x,10}$
ORC turbine (T2)	Energy balance	${\dot{W}}_{T2}={\dot{m}}_{12}\;\left(h_{12}-h_{13}\right)$
	Exergy balance	${\dot{E}}_{x,D,T2}={\dot{m}}_{12}\left(e_{x,12}-e_{x,13}\right)-{\dot{W}}_{T2}$
ORC condenser (C1)	Energy balance	${\dot{Q}}_{C1}={\dot{m}}_{12}\left(h_{13}-h_{14}\right)={\dot{m}}_{c1}\left(\;h_{c1,o}-h_{c1,i}\right)$
	Exergy balance	${\dot{E}}_{x,D,C3}={\dot{m}}_{20}\left(e_{x,20}-e_{x,21}\right)+{\dot{m}}_{C3}\left(e_{x,C3,i}-e_{x,C3,o}\right)$
ORC pump (P2)	Energy balance	${\dot{W}}_{P2}={\dot{m}}_{15}\;\left(h_{15}-h_{14}\right)$
	Exergy balance	${\dot{E}}_{x,D,P2}={\dot{m}}_{14}\left(e_{x,14}-e_{x,15}\right)+{\dot{W}}_{P2}$
Generator	Energy balance	${\dot{m}}_{CO2}h_{7}+{\dot{m}}_{sol}\;h_{22}={\dot{m}}_{CO2}\;h_{8}+{\dot{m}}_{r}\;h_{16}+\left({\dot{m}}_{sol}-{\dot{m}}_{r}\right)\;h_{23}$
	Exergy balance	${\dot{E}}_{x,D,gen}={\dot{m}}_{CO2}\left(e_{x,7}-e_{x,8}\right)+{\dot{m}}_{sol}e_{x,22}-\left({\dot{m}}_{sol}-{\dot{m}}_{r}\right)e_{x,23}-{{\dot{m}}_{r}e}_{x,16}$
ARC Condenser (C2)	Energy balance	${\dot{Q}}_{C2}={\dot{m}}_{r}\left(\;h_{16}-h_{17}\right)={\dot{m}}_{C2}\left(\;h_{C2,o}-h_{C2,i}\right)$
	Exergy balance	${\dot{E}}_{x,D,C2}={\dot{m}}_{r}\left(e_{x,16}-e_{x,17}\right)+{\dot{m}}_{C2}\left(e_{x,C2,i}-e_{x,C2,o}\right)$
Valve (V1)	Energy balance	$h_{17}=h_{18}$
	Exergy balance	${\dot{E}}_{x,D,V1}={\dot{m}}_{r}\left(e_{x,17}-e_{x,18}\right)$
Evaporator	Energy balance	${\dot{Q}}_{E}={m\dot{\;}}_{r}\;\left(h_{19}-h_{18}\right)$
	Exergy balance	${\dot{E}}_{x,D,E}={\dot{m}}_{r}e_{x,18}+{\dot{m}}_{E}e_{x,E,i}-{\dot{m}}_{r}e_{x,19}-{\dot{m}}_{E}e_{x,E,o}$
Valve (V2)	Energy balance	$h_{24}=h_{25}$
	Exergy balance	${\dot{E}}_{x,D,V2}=\left({\dot{m}}_{sol}-{\dot{m}}_{r}\right)\left(e_{x,24}-e_{x,25}\right)$
Absorber	Energy balance	${\dot{Q}}_{abs}=\left({\dot{m}}_{sol}-{\dot{m}}_{r}\right)h_{25}+{\dot{m}}_{r}\;h_{19}-{\dot{m}}_{sol}\;h_{20}={\dot{m}}_{abs}\left(\;h_{abs,o}-h_{abs,i}\right)$
	Exergy balance	${\dot{E}}_{x,D,abs}=\left({\dot{m}}_{sol}-{\dot{m}}_{r}\right)e_{x,25}+{\dot{m}}_{r}e_{x,19}-{\dot{m}}_{sol}e_{x,20}+{\dot{m}}_{abs}e_{x,abs,i}-{\dot{m}}_{abs}e_{x,abs,o}$
Solution pump (P3)	Energy balance	${\dot{W}}_{P3}={\dot{m}}_{sol}\;\left(h_{21}-h_{20}\right)$
	Exergy balance	${\dot{E}}_{x,D,P3}={\dot{m}}_{sol}\left(e_{x,20}-e_{x,21}\right)+{\dot{W}}_{P3}$
Solution Heat Exchanger	Energy balance	${\dot{m}}_{sol}\;h_{21}+\left({\dot{m}}_{sol}-{\dot{m}}_{r}\right)h_{23}=\left({\dot{m}}_{sol}-{\dot{m}}_{r}\right)h_{24}+{\dot{m}}_{sol}\;h_{22}$
	Exergy balance	${\dot{E}}_{x,D,SHE}=\left({\dot{m}}_{sol}-{\dot{m}}_{r}\right)\left(e_{x,23}-e_{x,24}\right)+{\dot{m}}_{sol}\left(e_{x,21}-e_{x,22}\right)$
Overall efficiency	Thermal	$\eta_{th,overall}=\frac{W_{net,s-CO2}+W_{net,ORC}+{\dot{Q}}_{E}}{{\dot{Q}}_{solar}}$
	Exergy	$\eta_{ex,overall}=\frac{W_{net,s-CO2}+W_{net,ORC}+{\dot{E}}_{x,E}}{{\dot{E}}_{x,solar}}$

## 5 Validation of system

Table 6, Table 7, Table 8, Table 9 plays a vital role in the validation process of our model, as it compares the simulation-generated data with data obtained from reputable research literature. The thermodynamic simulation of the solar central receiver, s-CO_2_ power cycle, ORC section, and ARC section has been validated using the results and data from Refs. [4,15,32,35]. We can find the simulation results and the results given in the literature to coincide with one another quite well, as shown in Table 6, Table 7, Table 8, Table 9. It is essential to note that some modifications have been implemented to the established model to conduct an appropriate comparison with the results from the literature.

**Table 6:** Comparison between obtained results of solar central receiver and data in Ref. [35].

Parameter	Ref. [35]	Present work	Deviation (%)
HTF	(67LiF, 33BeF_2_) Molten salt	(60NaNO_3_, 40KNO_3_) Molten salt	**-**
Energy efficiency of heliostat	75 %	75 %	0 %
Total heat received by the receiver	7500 kW	7500 kW	0 %
$T_{r}$	692°C	697.9°C	0.84 %
Energy efficiency of the receiver	76.44 %	90.33 %	15.38 %

**Table 7:** Comparison between obtained results of s-CO_2_ power cycle and data in Ref. [32].

Parameter	Ref. [32]	Present work	Deviation (%)
Inlet temperature of s-CO_2_ turbine	550°C	550°C	**-**
Inlet pressure of compressor	7.63 MPa	7.63 MPa	**-**
Outlet pressure of compressor	20 MPa	20 MPa	**-**
Inlet temperature of compressor	32°C	32°C	**-**
Thermal efficiency	36.87 %	37.18 %	0.83 %

**Table 8:** Comparison between obtained results of ORC cycle and data in Ref. [4].

Working Fluid	Parameter	Ref. [4]	Present work	Deviation (%)
Toluene	Condensation temperature	40°C	40°C	–
	Isentropic efficiency	85 %	85 %	–
	Thermal Efficiency	22.07 %	22.42 %	1.56 %

**Table 9:** Comparison between obtained results of ARC cycle and data in Ref. [15].

Parameter	Ref. [15]	Present study	Deviation
Generator temperature	90 °C	90 °C	–
Condenser temperature	35 °C	35 °C	–
COP	0.7316	0.7359	0.58 %

## 6 Simulation results and discussion

In this study, for a new configuration of the power-cooling cogeneration system, a thermodynamic investigation of the solar tower collector combined with a s-CO_2_ power cycle, an organic Rankine cycle employing three different working fluids, and single effect absorption refrigeration cycle has been performed. Based on the findings of using three different working fluids, including R123, R245fa, and toluene, as the working fluid for ORC, the following conclusions are drawn. In this research, a detailed analysis has been carried out, taking into account energy and exergy issues and the evaluation criteria of the system, such as the thermal and exergy efficiency of the cogeneration system, the power and cooling capacity assessment of the components under a wide range of operating conditions, will be examined. According to the current study, the effects of modifying the heliostat field area, solar irradiation, inlet temperature of s-CO_2_ turbine, evaporator temperature, and ORC condenser temperature on the combined cycle efficiencies of a new configuration of a power-cooling cogeneration system are investigated.

This research investigated the influence of heliostat field area on the energetic and exergetic performance of a power-cooling cogeneration system, using heliostat field areas ranging from 9000 to 11000 $m^{2}$. Fig. 3 depicts the change in the thermal and exergy efficiencies of a cogeneration system for power and cooling operating with three ORC working fluids, including R123, R245fa, and toluene, as a function of the heliostat field area used in the study.

**Fig. 3:** Variation of thermal and exergy efficiencies of proposed system with heliostat field area.

Following the trends shown in Fig. 3, it is discovered that the thermal and exergy efficiencies of the proposed power-cooling cogeneration systems for different ORC working fluids containing R123, R245fa, and toluene rise with an increase in the area of the heliostat field. Because as the heliostat field area is increased, the energy of solar heat input increases, and the outlet temperature of the fluid employed in the receiver also rises, which in turn results in increased energy input to the power and cooling cycles. Increasing the area of the heliostat field results in a notable rise in cycle power and cooling capacity due to the higher energy efficiency of the heliostat and receiver. As a consequence, the temperature of the working fluid increases significantly alongside the outlet temperature of molten salt. The study reveals that the cogeneration cycle exhibits a higher thermal efficiency than exergy efficiency. This is attributed to the lower exergy efficiency of the heliostat and receiver in comparison to their thermal efficiency, and that irreversibilities have occurred in the components of the cogeneration power cooling cycle.

Thermal and exergy efficiencies of power-cooling cogeneration systems are significantly influenced by changes in the working fluid of the ORC cycle due to the significant difference in their boiling points: (27.78 °C) for R123, (15.18 °C) for R245fa, and (110.6 °C) for toluene. More specifically, in the specified range of heliostat field area, it has been determined that a toluene-operated power-cooling cogeneration system has the highest thermal and exergy efficiencies due to its high critical temperature (318.6 °C), as it appeared differently concerning the lower critical temperatures of R123 (183.7 °C) and R245fa (154.01 °C). According to Fig. 3, the thermal efficiency of the proposed system increases from 46.49 % to 47.94 % for R245fa, from 47.72 % to 49.20 % for R123, and from 51.37 % to 52.97 % when toluene is used as a working fluid as the heliostat field area increases from 9000 to 11000 $m^{2}$.

Variations in the heliostat field area impact the power and refrigeration output of the system, as illustrated in Fig. 4. Increasing the heliostat field area within the range of 9000–11000 $m^{2}$ increases the power output and refrigeration output of the proposed system for the investigated working fluids. Many things are going on, but one big reason is that there are fewer heat losses in the receiver. For this reason, more heat is transferred to the heat transfer fluid, resulting in increased power and cooling production from the integrated system.

**Fig. 4:** Variation of turbine power and refrigeration output of proposed system with heliostat field area.

Based on all examined heliostat field areas, toluene shows the maximum turbine power output because of its high boiling and critical temperatures, whereas R245fa gives the lowest turbine power output since it has a low boiling and critical temperature. Additionally, varying the field area of the heliostat from 9000 to 11000 $m^{2}$ increases the power output from 2478 kW to 3123 kW for R245fa, from 2567 kW to 3235 kW for R123, and from 2830 kW to 3546 kW when toluene is used as the working fluid. Conversely, the examined ORC working fluid does not show any impact on the refrigeration output. However, as the heliostat area increases from 9000 to 11000 $m^{2}$, the refrigeration output rises from 873.9 kW to 1101 kW.

Fig. 5 illustrates the influence of solar irradiation on the thermal and exergy efficiencies of the power-cooling cogeneration system. It is found that the thermal and exergy efficiencies of the integrated system increases as solar irradiation increases from 900 to 1100 $W/m^{2}$. The heliostat's efficiency increases with higher solar irradiation, leading to greater energy capture and reflection onto the central receiver. Moreover, elevated solar irradiation also raises the surface temperature of the receiver, providing an additional advantage. However, because of the small margin, emissive and convective heat losses are minimized, which is a significant benefit because the temperature of molten salt at the outlet is dependent on it. Due to the significant quantity of heat energy imparted to the heat transfer fluid, an elevation in surface temperature shall occur, leading to a subsequent increase in the temperature of the molten salt and eventually the CO_2_ flowing into the s-CO_2_ turbine. Increasing the CO_2_ fluid temperature that goes into the s-CO_2_ turbine will result in the s-CO_2_ turbine producing more power and hence increasing the cooling capacity. This figure represents the remarkable performance of the proposed system for toluene as an ORC working fluid, whereas the R245fa represents the lowest performance of the proposed system.

**Fig. 5:** Impact of Solar Irradiation on the thermal and exergy efficiency of proposed system.

Fig. 6 illustrates the influence of solar irradiation on the power output and refrigeration output of a proposed power-cooling cogeneration system with three ORC working fluids. This figure demonstrates that when the intensity of solar irradiation increases, the power and refrigeration output increase. Because of reduction in receiver loss and, as a result, an improvement in receiver efficiency, which results in a higher amount of energy delivered to the prime mover of the proposed system. As a result, the proposed system exhibits an increase in power output, generated from the s-CO2 and ORC turbine, as well as an increase in cooling capacity produced by the ARC cycle. Toluene has the highest turbine power output (from 2859 kW to 3545 kW) of all the investigated solar irradiation (from 900 to 1100 $W/m^{2}$), while R245fa has the lowest turbine power output (from 2503 kw to 3104 kW). Furthermore, as the solar irradiation increases from 900 to 11000 $W/m^{2}$, the refrigeration output also increases from 888.2 kW to 1095 kW for all the ORC working fluids studied. This is due to the fact that the examined ORC working fluid does not have any effect on the refrigeration output.

**Fig. 6:** Impact of the solar irradiation on the turbine power output and refrigeration output of proposed system.

Fig. 7 exhibits the impact of s-CO_2_ turbine inlet temperature on the power and refrigeration output of the cogeneration system employing different ORC operating fluids such as R123, R245fa, and toluene. This figure clearly defines that the power output produced by the s-CO_2_ turbine rise with the rise in inlet temperature of the s-CO_2_ turbine. An increase in inlet temperature of a s-CO_2_ turbine from 450 °C to 750 °C causes a rise in the enthalpy difference within the s-CO_2_ turbine, resulting in an increase in power output. Fig. 7 demonstrates that the ORC turbine power output and refrigeration output both show a minor decline with an increase in turbine inlet temperature. The reduction in power output of the s-CO2 cycle and cooling capacity of the ARC cycle can be attributed to the reduction in mass flow rate within the s-CO2 cycle and the lower temperature of exhaust heat from the s-CO_2_ turbine, which is harnessed for driving both the ORC cycle and ARC cycle.

**Fig. 7:** Effect of s-CO_2_ turbine inlet temperature on the power and refrigeration output of the proposed system.

According to Fig. 8, increasing the s-CO_2_ turbine inlet temperature impacts the thermal and exergy efficiencies of the proposed power-cooling cogeneration system when three different ORC operating fluids are employed. This figure clearly defines that the thermal and exergy efficiencies of the proposed system increase with the rise in turbine inlet temperature from 450 °C to 750 °C. This is due to the larger increment in s-CO2 cycle power output relative to the decreases in ORC turbine power output and refrigeration output, resulting in a rise in efficiencies of the system. It observes that as the temperature of the turbine inlet increases, the proposed cogeneration system achieves the maximum thermal and exergy efficiencies using toluene as the working fluid, whereas R245fa achieves the lowest thermal and exergy efficiencies.

**Fig. 8:** Effect of s-CO_2_ turbine inlet temperature on the thermal and exergy efficiencies of the proposed system.

The influence of varying the evaporator temperature of ARC cycle on the thermal and exergy efficiencies of the cogeneration system was carefully monitored and is depicted in Fig. 9. We can see that the thermal efficiency of the cogeneration system improves when the evaporator temperature is varied from 270 K to 286 K. The reason for this phenomenon is the increase in heat input into the evaporator that occurs when the evaporator temperature rises. Toluene was found to have the highest thermal efficiency of all of the ORC working fluids studied. Furthermore, the thermal efficiency of the proposed system rises from 47.27 % to 47.42 % for R245fa, from 48.51 % to 48.67 % for R123 and from 52.24 % to 52.39 % when toluene is employed as an operating fluid at a given evaporator temperature of ARC cycle. Further, it has been discovered that the exergy efficiency of the proposed cogeneration system drops a little when the temperature of the evaporator in ARC cycles rises. This is because the evaporator temperature is an integral part of the exegetic formulation, as the numerator is expressed as ${\dot{Q}}_{Evap}\left(1-\frac{T_{o}}{T_{Evap}}\right)$. As a result of this relationship, the heat output from the evaporator increases when the evaporator temperature rises, reducing the exergy efficiency of the ARC cycle. It is noticed that increasing the evaporator temperature of the ARC cycle declines the exergy efficiency of the proposed system from 41.43 % to 40.57 % for R245fa, from 42.85 % to 41.99 % in the case of R123, and from 47.11 % to 46.25 % for toluene.

**Fig. 9:** Variation of evaporator temperature of ARC cycle on the thermal and exergy efficiency of proposed system.

Fig. 10 depicts the influence of increasing the condenser temperature of the ORC cycle on the thermal and exergy efficiencies of the proposed power cooling cogeneration system. From the figure, we can see that the thermal and exergy efficiencies of the cogeneration system decline significantly as the temperature of the ORC condenser is raised. Because of the lower enthalpy drop in the turbine, the thermal efficiency of the cogeneration system is reduced. According to the thermophysical properties of organic fluids, increasing the condenser temperature results in a rise in exergy input and exergy destruction in the condenser. The investigation revealed that increasing the temperature of the ORC condenser from 30 °C to 42 °C caused a decline in the thermal efficiency from 47.66 % to 46.91 % when R245fa was used as the working fluid and from 48.90 % to 48.16 % when R123 was used, and from 52.57 % to 51.97 % in the case of toluene working fluid. The results indicate that among all the ORC condenser temperatures tested, toluene has the highest performance, while R245fa has the lowest performance.

**Fig. 10:** The impact of condenser temperature of ORC cycle on the thermal and exergy efficiencies of the proposed system.

Fig. 11 presents a comprehensive breakdown of exergy destruction rate in each subsystem for three working fluids within the proposed system. This exergy analysis is crucial in enhancing comprehension of the irreversibility underlying the solar driven power-cooling cogeneration cycle. After conducting a detailed exergy analysis, it was determined that when the system is subjected to a 100 % exergy destruction rate for each individual subsystem, the analysis revealed that the solar tower receiver accounts for the highest percentage of exergy destruction rate within system (73.24 %) followed by the s-CO2 cycle (11.72 %), ARC cycle (11.02 %), and ORC cycle (4.02 %) when utilizing toluene as the working fluid. The solar tower receiver is known to yield significant exergy dissipation due to the high temperature (high quality) losses of heat from the receiver to the surrounding environment. Hence, it is imperative to direct additional research efforts towards the enhancement of the design and the reduction of losses in the solar tower receiver. Furthermore, when utilizing R123 as the working fluid, the solar tower receiver contributes to the most significant proportion of exergy destruction rate within system (67.80 %), with the ORC cycle accounting for 11.08 %, the s-CO2 cycle for 10.92 %, and the ARC cycle for 10.20 %. Similarly, when R245fa is used as the working fluid, the solar tower receiver contributes to the highest percentage of exergy destruction rate within system (66.19 %), followed by the ORC cycle (13.25 %), s-CO2 cycle (10.60 %), and ARC cycle (9.96 %).

**Fig. 11:** Breakdown of exergy destruction rate in each subsystem for three working fluids within the proposed system.

## 7 Conclusion

This study performed a thermodynamic analysis on a configuration of a solar tower collector combined with s-CO_2_, ORC, and ARC cycles for cogeneration of power and cooling. The proposed cogeneration system employs molten salt as a medium for heat transfer within the collector. In this study, power is produced by employing s-CO_2_ and ORC cycles using three different working fluids: R123, R245fa, and toluene. Additionally, the ARC cycle is used to produce refrigeration output. This research conducted the energetic and exergetic assessment of the components under various operating conditions and parameters, including heliostat field area, solar irradiation, evaporator temperature, inlet temperature of s-CO_2_ turbine, and condenser temperature of ORC are altered to ascertain their influence on power and cooling output, as well as the thermal and exergy efficiencies of the proposed system. The primary conclusions drawn from the obtained results and computational data may be summarized as follows:

• All three ORC working fluids studied have shown that toluene produces the highest turbine power, resulting in the highest overall efficiency, whereas R245fa produces the lowest performance.
• The thermal and exergy efficiency of the proposed system increases from 46.49 % to 47.94 % and 40.25 %–41.5 % for R245fa, from 47.72 % to 49.20 % and 41.65 %–42.94 % for R123, and from 51.37 % to 52.97 % and 45.82 %–47.25 % when toluene is used as a working fluid as the heliostat field area increases from 9000 to 11000 $m^{2}$.
• The performance of the proposed cogeneration system increase as the solar irradiation rises. It is noted that the refrigeration capacity improved from 882.8 kW to 1095 kW in response to a rise in solar irradiation from 900 to 1100 $W/m^{2}$.
• As the inlet temperature of s-CO_2_ turbine varied from 450 °C to 750 °C and toluene was employed as a working fluid, thermal efficiency increased from 47.96 % to 58.73 %, and exergy efficiency increased from 44.39 % to 55.26 %.
• Further, the thermal efficiency of the system rises from 47.27 % to 47.42 % for R245fa, from 48.51 % to 48.67 % for R123, and from 52.24 % to 52.39 % when toluene is employed as a working fluid at a given ARC evaporator temperature.
• The energetic and exergetic performance of the cogeneration system decreased marginally when the temperature of the ORC condenser increased from 30 °C to 42 °C. With all investigated ORC condenser temperatures, toluene achieves the highest performance, while R245fa obtains the lowest performance.
• The primary contributor of exergy destruction rate in the proposed system was determined to be the solar tower receiver, contributing 73.24 %, 67.80 %, and 66.19 % to the total for the toluene, R123, and R245fa working fluids, respectively.

Additional comprehensive research and economic evaluation are required to fully evaluate the practicality and sustainability of the solar tower collector-based integrated system developed for simultaneous production of power and cooling. Given the inherently intermittent and variable nature of solar energy, it is strongly advised that forthcoming studies investigate and incorporate diverse energy storage techniques suitable for the existing system.

## CRediT authorship contribution statement

**Mohd Asjad Siddiqui:** Writing – review & editing, Writing – original draft, Validation, Supervision, Investigation, Formal analysis, Data curation, Conceptualization. **Ibrahim Alsaduni:** Supervision, Project administration, Funding acquisition.

## Data availability statement

Data will be made available on request.

## Declaration of Competing Interest

The authors declare that they have no known competing financial interests or personal relationships that could have appeared to influence the work reported in this paper.

## Nomenclature

**Symbols**
A: Area $\left(m^{2}\right)$
$C_{p}$: Specific heat (kJ/kg K)
$\dot{E_{x}}$: Rate of exergy (kW)
$e_{x}$: Specific exergy (kJ/kg)
$F_{r}$: View factor
h: Specific enthalpy (kJ/kg)
k: Thermal conductivity (W/m K)
$\dot{m}$: Rate of flowing mass (kg/s)
$\dot{Q}$: Rate of heat transfer (kW)
s: Entropy per unit mass (kJ/kg K)
T: Temperature (K)
$\dot{W}$: Work output (kW)

**Greek symbols**
η: Efficiency (%)
ε: Average emissivity
σ: Stefan–Boltzmann constant
χ: Reflectivity

**Subscript**
abs: Absorber; absorbed
ap: Aperture
C1: ORC condenser
C2: Condenser of ARC
CR: Central receiver
em: Emissive
Des: Desorber
D: Destruction
E: Evaporator
H: Heliostat
i: Inlet
ms: Molten salt
o: Outlet
P1: Molten salt pump
P2: Pump of ORC cycle
P3: Solution pump of ARC
r: Refrigerant; receiver
sol: Solution

**Abbreviations**
s-CO_2_: Supercritical carbon-dioxide
ORC: Organic Rankine cycle
ARC: Absorption refrigeration cycle
